# Nutrition status mediates the association between cognitive decline and sarcopenia

**DOI:** 10.18632/aging.202672

**Published:** 2021-03-10

**Authors:** Xiaolei Liu, Xin Xia, Fengjuan Hu, Lisha Hou, Shuli Jia, Yixin Liu, Linghui Deng, Yan Zhang, Wanyu Zhao, Gongchang Zhang, Jirong Yue, Birong Dong

**Affiliations:** 1 National Clinical Research Center for Geriatrics, West China Hospital, Sichuan University, Chengdu, Sichuan Province, China; 2 Geriatric Health Care and Medical Research Center, Sichuan University, Chengdu, Sichuan Province, China

**Keywords:** sarcopenia, nutrition status, cognitive decline, mediator

## Abstract

In this study, we investigated whether nutrition status mediates the relationship between cognitive decline and sarcopenia. Sarcopenia was assessed in 4023 community-dwelling older adults from West China using the AWGS 2014 diagnostic criteria. Cognitive function and nutrition status were assessed using the 10-item Short Portable Mental Status Questionnaire (SPMSQ) and Mini Nutrition Assessment-Short Form (MNA-SF) scale, respectively. Mediation model regression analysis demonstrated that nutrition status was negatively associated with sarcopenia (β = -0.521; 95% CI: -0.583 to -0.459). The indirect effects of cognitive decline on sarcopenia were significant after adjusting for age, sex, and ethnicity (β = 0.015; 95% CI: 0.012 to 0.017), but the direct effects of cognitive decline on sarcopenia were not statistically significant after adding nutrition status as a parameter in the mediation model analysis (β = -0.001; 95% CI: -0.008 to 0.005). Structural equation model (SEM) framework pathway analysis confirmed the association between nutrition status, cognitive decline, and sarcopenia. These findings demonstrate that the negative effects of cognitive decline on sarcopenia were mediated by nutrition status. We therefore postulate that maintaining a good nutrition status delays the negative effects of cognitive decline on sarcopenia in older adults.

## INTRODUCTION

Sarcopenia is defined as age-related loss of skeletal muscle mass and strength, and is associated with significant disability and morbidity among the elderly [1, 2]. The prevalence of sarcopenia varies among different populations worldwide because of differences in the diagnostic criteria. The prevalence of sarcopenia was 21.3% in males and 13.8% in females according to the AWGS 2019 criteria, which was used to analyze 2123 ambulatory community-dwelling older adults between 70 and 84 years of age in the nationwide Korean Frailty and Aging Cohort Study (KFACS) [3]. The meta-analysis by Shafiee et al. included 58404 study subjects and showed that the world-wide prevalence of sarcopenia was 10% (95% CI: 8-12%) in men and 10% (95% CI: 8-13%) in women [4]. Another meta-analysis by Pacifico et al. showed that sarcopenia was highly prevalent among individuals with cardiovascular diseases, dementia, diabetes mellitus, and respiratory diseases [5]. For example, prevalence of sarcopenia was 26.4% (95% CI: 13.6–44.8%) in individuals with dementia compared to 8.3% (95% CI: 2.8–21.9%) in those without dementia [5].

The risk factors associated with sarcopenia include old age, smoking, malnutrition, lower physical activity, low serum albumin levels, and vitamin D deficiency [6]. Malnutrition increased the risk of sarcopenia by at least 13 fold in elderly adults [6]. Hsu et al. performed a long term cohort study in older men and showed that the risk of malnutrition was significantly associated with 3-year cognitive decline (OR: 2.07, 95% CI: 1.05-4.08, P =0.036) [7]. Kimura et al. studied older women with mild cognitive impairment and early stage Alzheimer’s disease, and showed that malnutrition was common in older adults with mild cognitive decline [8]. This suggested a potential association between cognitive decline, malnutrition, and sarcopenia. These findings also suggested that malnutrition was a key factor that could negatively impact both cognitive decline and sarcopenia. A recent study by Perez-Sousa et al. showed that the negative effect of sarcopenia on daily living activities was mediated by gait speed, thereby suggesting that physical exercise could maintain gait speed and delay sarcopenia in older individuals [9]. Therefore, in this study, we used mediation analysis to determine if nutrition status mediated the effects of cognitive decline on sarcopenia.

## RESULTS

### Sarcopenia is significantly associated with cognitive decline and nutrition status

Figure 1 shows the mediation model with ‘M’ as the mediator variable (nutrition status), ‘X’ as antecedent variable (cognitive decline), and ‘Y’ as the outcome variable (sarcopenia). The differences in various clinical characteristics between sarcopenia and non-sarcopenia groups are shown in Table 1. The overall prevalence of sarcopenia in our study was 18.2% based on the AWGS 2014 diagnostic criteria. The prevalence of sarcopenia was 21.5% in men and 16.4% in women. Older study subjects showed higher prevalence of sarcopenia compared to the younger subjects (50-59yrs 9.1%, 60-69yrs 18.3%, 70-79yrs 39.0%, 80+yrs 67.1%). The prevalence of sarcopenia was higher among individuals belonging to the Yi ethnicity group than other ethnicity groups. The prevalence of sarcopenia was higher among smokers and individuals with poor sleep quality. Individuals with lower education as well as lower weight, height and BMI showed increased prevalence of sarcopenia. Moreover, our study showed that both cognitive decline and malnutrition were significantly associated with sarcopenia, and showed a dosage effect (prevalence of sarcopenia: mild cognitive decline, 17.3%; moderate cognitive decline, 25.5%; severe cognitive decline, 42.9%; malnutrition risk, 24.6%; malnutrition 54.9%).

**Figure 1:** **Statistical mediation simple diagram.**

**Table 1:** Sample characteristics stratified by sarcopenia status (N=4023).

**Sample characteristics**	**Total n=4023**	**Sarcopenia n=734(18.2)**	**Non-sarcopenia n=3289(81.8)**	**p value**
**Male, n(%)**	1477(36.7)	317(21.5)	1160(78.5)	<.001
**Female, n(%)**	2546(63.3)	417(16.4)	2129(83.6)	<.001
**Age, mean(SD)**	62.2(8.2)	67.6(8.7)	61.0(7.5)	<.001
**Male, age, mean(SD)**	61.4(8.1)	68.9(8.1)	62.2(7.6)	<.001
**Female, age, mean(SD)**	63.7(8.2)	66.7(9.1)	60.3(7.4)	<.001
**Age group, n(%)**				
**50-59**	1789(44.5)	162(9.1)	1627(90.9)	<.001
**60-69**	1559(38.8)	285(18.3)	1274(81.7)	
**70-79**	590(14.7)	230(39.0)	360(61.0)	
**80 +**	85(2.1)	57(67.1)	28(32.9)	
**Ethnic group, n(%)**				
**Han**	1773(44.1)	377(21.3)	1396(78.7)	<.001
**Zang**	1025(25.5)	179(17.5)	846(82.5)	
**Qiang**	987(24.5)	112(11.3)	875(88.7)	
**Yi**	175(4.3)	51(29.1)	124(70.9)	
**others**	63(1.6)	15(23.8)	48(76.2)	
**Educational level, n(%)**				
**No formal education**	1155(28.7)	265(22.9)	890(77.1)	<.001
**Elementary school**	1386(34.5)	263(19.0)	1123(81.0)	
**Middle school**	894(22.2)	128(14.3)	766(85.7)	
**High school and above**	588(14.6)	78(13.3)	510(86.7)	
**Occupation**				
**White-collar worker**	366(9.1)	56(15.3)	310(84.7)	<.001
**Service worker**	217(5.4)	45(20.7)	172(79.3)	
**Industrial workers**	362(9.0)	54(14.9)	308(85.1)	
**Soldier**	38(0.9)	9(23.7)	29(76.3)	
**Farmers**	2648(65.8)	523(19.8)	2125(80.2)	
**Businessman**	174(4.3)	16(9.2)	158(90.8)	
**Others**	218(5.4)	31(14.2)	187(85.8)	
**Smoking status, n(%)**				
**Yes**	707(17.6)	173(24.5)	534(75.5)	<.001
**No**	3315(82.4)	560(16.9)	2755(83.1)	
**Drinking alcohol status, n(%)**				
**Yes**	1036(25.8)	182(17.6)	854(82.4)	.509
**No**	2986(74.2)	552(18.5)	2434(81.5)	
**Drinking tea status, n(%)**				
**Yes**	1942(48.3)	393(18.9)	1602(81.1)	.249
**No**	2078(51.7)	340(17.5)	1685(82.5)	
**Sleeping quality, n(%)**				
**Yes**	1888(46.9)	373(50.8)	1515(46.1)	.020
**No**	2135(53.1)	361(49.2)	1774(53.9)	
**Disease comorbidity, n(%)**				
**Yes**	2950(73.3)	556(18.8)	2394(81.2)	.101
**No**	1073(26.7)	178(16.6)	895(83.4)	
**Depression status, n(%)**				
**Yes**	724(18.0)	150(20.7)	574(79.3)	.057
**No**	3299(82.0)	584(17.7)	2715(82.3)	
**Anxiety status, n(%)**				
**Yes**	779(19.4)	139(17.8)	640(82.2)	.746
**No**	3244(80.6)	595(18.3)	2649(81.7)	
**Anthropometry, mean(SD)**				
**Weight (kg)**	62.2(11.2)	51.9(8.2)	64.5(10.5)	<.001
**Height (cm)**	156.4(8.1)	152.9(8.1)	157.2(7.9)	<.001
**BMI (kg/m**^2^**)**	25.3(3.8)	22.0(2.7)	26.1(3.6)	<.001
**Gait speed (m/s)**	0.86(0.27)	0.75(0.27)	0.88(0.26)	<.001
**Grip strength (kg)**	22.3(8.7)	17.9(6.9)	23.2(8.7)	<.001
**SMI (kg/m**^2^**)**	6.6(0.9)	5.7(0.7)	6.8(0.9)	<.001
Cognitive score*	1 (0-2)	1(0-2)	1(0-2)	<.001
**Mild cognitive decline**	3577(88.9)	619(17.3)	2958(82.7)	<.001
**Moderate cognitive decline**	439(10.9)	112(25.5)	327(74.5)	
**Severe cognitive decline**	7(0.2)	3(42.9)	4(57.1)	
Nutrition status score*	11(10-12)	11(10-12)	10(9-11)	<.001
**Normal**	1725(42.9)	142(8.2)	1583(91.8)	<.001
**Malnutrition risk**	2207(54.9)	542(24.6)	1665(75.4)	
**Malnutrition**	91(2.3)	50(54.9)	41(45.1)	

Note. Means ± standard deviation was shown. Others=other nationalities including Zhuang, Manchu, Hui, Mongolia, Tujia nationalities. Data are shown using % or mean (standard deviation). P values were calculated with chi-squared tests and Student's t tests for categorical and continuous variables, respectively.* These variables are presented as median (interquartile range).

### Nutrition status mediates the association between cognitive decline and sarcopenia

Table 2 shows the association between cognitive scores of the study subjects and sarcopenia. The regression analysis demonstrated significant association between cognitive score and sarcopenia, and this association was independent of age, gender, ethnicity, life style, sleep quality, depression, anxiety, and chronic disease comorbidity. However, regression analysis showed that the association between cognitive score and sarcopenia was not statistically significant when the model included nutrition score as a parameter (p=0.7). This suggested that nutrition status may influence the association between cognitive decline and sarcopenia.

**Table 2:** Associations between cognitive status and sarcopenia in older adults.

**Outcome variable**		**OR**	**P-value**	**95% CI**
	**sarcopenia**			
**Model 1**	**Cognitive score**	1.162	<0.001	1.111 to 1.215
	**gender**	1.323	0.002	1.113 to 1.572
	**age**	1.096	<0.001	1.085 to 1.108
	**Ethnic groups**	1.343	0.001	1.137 to 1.587
**Model 2**	**Cognitive score**	1.157	<0.001	1.054 to 1.187
	**gender**	1.236	0.123	0.953 to 1.497
	**age**	1.096	<0.001	1.085 to 1.108
	**Ethnic groups**	1.290	0.003	1.088 to 1.530
	**Drinking**	0.743	0.006	0.601 to 0.920
	**Smoking**	1.537	0.001	1.202 to 1.965
	**Drinking tea**	0.982	0.839	0.823 to 1.172
	**Sleep quality**	1.064	0.469	0.899 to 1.259
**Model 3**	**Cognitive score**	1.149	<0.001	1.098 to 1.203
	**gender**	1.245	0.047	1.003 to 1.545
	**age**	1.097	1.097	1.085 to 1.108
	**Ethnic groups**	1.313	0.002	1.105 to 1.559
	**Drinking**	0.740	0.006	0.598 to 0.916
	**Smoking**	1.527	0.001	1.194 to 1.953
	**Drinking tea**	0.994	0.943	0.832 to 1.186
	**Sleep quality**	1.043	0.628	0.879 to 1.238
	**Chronic disease**	1.227	0.036	1.014 to 1.486
	**depression**	1.211	0.083	0.975 to 1.505
	**anxiety**	0.977	0.977	0.782 to 1.219
**Model 4**	**Cognitive score**	0.988	0.700	0.930 to 1.050
	**gender**	1.176	0.177	0.929 to 1.487
	**age**	1.097	<0.001	1.085 to 1.110
	**Ethnic groups**	1.427	<0.001	1.184 to 1.718
	**Drinking**	0.775	0.029	0.616 to 0.975
	**Smoking**	1.369	0.021	1.048 to 1.789
	**Drinking tea**	1.117	0.262	0.920 to 1.357
	**Sleep quality**	1.019	0.846	0.846 to 1.226
	**Chronic disease**	1.149	0.187	0.935 to 1.412
	**depression**	1.088	0.492	0.855 to 1.384
	**anxiety**	0.931	0.567	0.730 to 1.188
	**Nutrition status**	0.601	<0.001	0.564 to 0.640

Note. Multiple logistic regression analysis between cognitive score and sarcopenia. Model 1 = adjusted by gender, age, and ethnic group; Model 2 = adjusted by Model 1 +life styles (smoking, drinking alcohol and drinking tea), sleep quality; Model 3 = adjusted by Model 2+chronic disease comorbidity, depression and anxiety. Model 4= adjusted by Model 3+nutrition status.

We then performed mediation model analysis to determine if nutrition status mediated the effects of cognitive decline on sarcopenia. As shown in Figure 2, regression analysis showed that cognitive decline correlated with worse nutrition status (β = -0.235; 95% CI: -0.265 to -0.206), and nutrition status score showed direct association with sarcopenia (β = -0.521; 95% CI: -0.583 to -0.459). The indirect effects of cognitive decline on sarcopenia were statistically significant (β = 0.015; 95% CI: 0.012 to 0.017), but the direct effects of cognitive decline on sarcopenia were not statistically significant (β = -0.001; 95% CI: -0.008 to 0.005). However, the total effect of cognitive decline on sarcopenia was statistically significant (β = 0.013; 95% CI: 0.006 to 0.020). This suggested that nutrition status mediates the association between cognitive decline and sarcopenia.

**Figure 2:** **Nutrition status as mediator of the effect of cognitive decline on sarcopenia.**

### SEM pathway analysis confirms the association between sarcopenia, cognitive decline, and nutrition status

We then performed path analysis using the structural equation model (SEM) framework. As shown in Figure 3, SEM pathway analysis showed that the correlation between cognitive decline and sarcopenia was positive (SEM co-efficient: 0.02), but, the association between cognitive decline and nutrition status was negative (SEM co-efficient: -0.26). Moreover, the correlation between nutrition status and sarcopenia was negative (SEM coefficient: -0.29). Furthermore, age, gender and ethnicity showed different positive estimate coefficients compared to cognitive decline, nutrition status and sarcopenia. The P value of the entire pathway in the SEM structure model was statistically significant. These results further confirmed the association between sarcopenia, nutrition status, and cognitive decline.

**Figure 3:** **A path analysis using the SEM framework.** Note. This framework shows that the estimate coefficient of cognitive decline to sarcopenia was 0.02, having a positive influence. The estimate coefficient of cognitive decline to nutrition status was -0.26, having a negative influence. The estimate coefficient of nutrition status to sarcopenia was -0.29, having a negative influence. Age, gender and ethnic groups have different estimate coefficient to the cognitive decline. nutrition status and sarcopenia. P value of all the pathway shown in framework were significant.

## DISCUSSION

To the best of our knowledge, this is the first study to evaluate the mediating role of nutrition status in the relationship between cognitive decline and sarcopenia. Our study demonstrates that nutrition status mediates the effects of cognitive decline on sarcopenia in older adults. Older adults with early characteristics of cognitive decline and better nutrition status are less likely to develop sarcopenia. Therefore, better nutrition status ameliorates negative effects of cognitive decline on sarcopenia.

The overall prevalence of sarcopenia in our study population was 18.2% based on the AWGS 2014 diagnostic criteria. This was higher than the previously published meta-analysis by Tian et al., which reported a sarcopenia prevalence of 11% in community-dwelling Chinese individuals aged 60 years and older [10]. The higher prevalence of sarcopenia in this study may be due to several reasons. Firstly, the higher prevalence of sarcopenia might be related to the poor economic status of our study subjects in rural west China. Dorosty et al. reported that the odd risk of sarcopenia was more likely 0.97 times higher in the lower socioeconomic class compared to those in the middle- and high-income classes [11]. Secondly, most of the study subjects in our study were farmers who lived alone and showed poor sleep quality and lower education levels. These factors are well recognized risk factors of sarcopenia [6]. Thirdly, the participants in our study belonged to various ethnicity groups, including Zang, Qiang, Yi and others. Most of them lived in huge mountainous regions and vast grasslands where medical resources were poor. Moreover, people living in these areas did not pay attention to their health. As a result, chronic disease burden was high in these ethnicity groups and potentially contributed to the higher prevalence of sarcopenia. It is also plausible that the AWGS 2014 diagnostic criteria were not optimal for this group of study subjects. Therefore, in the future, specific cutoff points based on the local factors need to be taken into account while diagnosing sarcopenia. Our study included 4500 participants with 2873 women and 1627 men. The prevalence of sarcopenia in men was higher than women in our study (21.5% vs. 16.4%). Previous studies have shown that women are more prone to sarcopenia than men because of hormonal levels such as estrogen, androgen, cortisol and so on [12]. However, our study was consistent with a previous meta-analysis by Tian et al., which reported that the prevalence of sarcopenia in elderly Chinese men was 1.5 times higher than women [10]. Another possible reason for this trend could be that the mean age of men in our study was higher compared to the women (63 years vs. 61 years).

Our results clearly show that smokers and individuals with poor sleep quality show higher prevalence of sarcopenia. Several epidemiological studies have shown increased prevalence of sarcopenia in elderly long-time smokers [10]. The components of cigarette smoke (CS) increase oxidative stress either directly or by activation of nicotinamide adenine dinucleotide phosphate (NADPH) oxidases (NOXs) in the skeletal muscle tissues that promote phosphorylation of p38 MAPK and activation of NF-kB, which subsequently upregulate muscle-specific E3 ubiquitin ligases that cause muscle degradation [13]. A recent meta-analysis showed that prevalence of sarcopenia was higher in older adults with inadequate sleep [14]. Individuals with poor sleep quality show elevated levels of cortisol, a catabolic hormone that promotes protein degradation, and lower levels of IGF-1, an anabolic hormone that promotes protein synthesis, thereby causing increased muscle degradation and loss of muscle mass [15, 16]. Moreover, sleep deprived individuals show higher circulating levels of c-reactive protein (CRP), which is associated with muscular atrophy [2].

The relationship between cognitive decline and sarcopenia is complex and bidirectional, and most likely regulated by several mechanisms. Firstly, older adults with cognitive decline demonstrate reduced physical activity and dietary intake, which triggers excessive muscle loss and accelerates sarcopenia [17]. Secondly, increased levels of pro-inflammatory factors interleukin-6 (IL-6) and tumor necrosis factor-α (TNF-α) are reported in patients with sarcopenia [18] and Alzheimer's cognitive impairment [19]. Thirdly, products of oxidative and nitrosative stress accumulate during aging and promote cognitive impairment [20]. Excessive oxidative stress alters the homeostatic balance between protein synthesis and breakdown, induces mitochondrial dysfunction and apoptosis, all of which promotes age-related muscle atrophy and eventually sarcopenia [21]. Furthermore, aberrant changes in the levels and activity of neurotransmitters in the central nervous system and inadequate distribution of oxygen to the brain in cognitive impaired individuals reduce muscle activity and contribute to sarcopenia [22].

In our study, we demonstrated that nutrition status is a critical mediator of the relationship between cognitive decline and sarcopenia. The mediation model and SEM framework pathway analyses showed that indirect effects of cognitive decline on sarcopenia were significant (β = 0.015; 95% CI: 0.012 to 0.017) after adjusting for age, sex, and ethnicity, but the direct effects of cognitive decline on sarcopenia were not statistically significant when analyzed in combination with nutrition status (β = -0.001; 95% CI: -0.008 to 0.005). This suggested that nutrition status mediated the association between cognitive decline and sarcopenia. Besides, SEM framework pathway analysis confirmed the results of the mediation analysis. There are several plausible explanations for our findings. Firstly, there is a close relationship between cognitive decline, nutrition status, and sarcopenia. Kang et al. demonstrated that nutritional deficiency in early life was associated with age-related cognitive decline [23]. Assis et al. reported that early identification of malnutrition through nutritional assessments helped prevent cognitive impairment in many cases [24]. Moreover, malnutrition promotes chronic low-grade inflammation, as observed in the malnutrition-inflammation-complex syndrome (MICS) [25]. Therefore, malnutrition promotes cognitive decline, which further increases the risk of sarcopenia and affects the daily living activities in the elderly [24]. Secondly, the earliest signs of cognitive decline include reduced ability to prepare food, forgetting to eat, and inability to access food, all of which can impair oral food intake and result in malnutrition [26]. Thirdly, our findings confirm previous reports that show that individuals with sarcopenia are associated with worse nutritional status [27] and cognitive decline [28]. Consequently, improving nutrition levels in older adults can maintain muscle mass and prevent sarcopenia. Cerri et al. reported that sarcopenia was highly prevalent in a population of hospitalized elderly individuals that were malnourished or at risk of malnutrition and was associated with increased risk of short-term mortality [29]. Malnutrition is characterized by muscle atrophy and overall decline in body muscle mass [30]. Skeletal muscle tissue constitutes majority of the protein-rich lean body mass and its atrophy significantly reduces muscle strength as shown by reduced hand grip strength (HGS) and muscle strength [31].

There are several limitations in this study. For example, smaller sample size, characteristics of the study population such as most participants in our study were relatively healthy, study design was cross-sectional study, and type of sampling did not cover all the cities in west China. All of these are potential source of bias. Another limitation of our study is that we used BIA alone to assess body composition of the study subjects. EWGSOP reviewed several tools to evaluate body composition and identified dual-energy X-ray absorptiometry and BIA as the most suitable techniques to clinically determine body composition of our study subjects. However, we conducted a centralized investigation and not a household survey. Hence, most of the participants who came to the site of investigation on their own were relatively healthy. This may have affected the actual determination of sarcopenia prevalence in the study community. However, we analyzed sufficient samples that allowed evaluation of regression models after optimally adjusting for multiple confounding factors. Moreover, the results of our study were similar to previous reports, thereby demonstrating robustness of our analysis.

In conclusion, our study demonstrated that the relationship between cognitive decline and sarcopenia was mediated by nutrition status. Therefore, our study suggests that improved nutrition status in older adults with cognitive decline can delay or counteract sarcopenia.

## MATERIALS AND METHODS

### Study design and data collection

We performed this analysis using data from the West China Health and Aging Trend (WCHAT) study, which was conducted in accordance with the 1964 Declaration of Helsinki guidelines and its later amendments. The research was approved by the Ethical Review Committee of West China Hospital (Committee reference number: 2017(445); Registration number: ChiCTR 1800018895). Previous reports have published details of the surveys used to generate this data [27, 28, 32]. The data was collected from Yunnan, Guizhou, Sichuan, and Xinjiang provinces in West China. The enrolled participants were 50 years and older. We obtained written and signed informed consent from all participants. The base-line response rate derived from multi-stage cluster sampling was 50.2%. Initially, we recruited 7536 community-dwelling multi-ethnic residents for this study. Among these, 4500 participants were eligible for further analysis of sarcopenia characteristics based on the bioelectrical impedance analysis (BIA). Finally, 4023 participants were included for analysis after excluding 467 participants for not completing nutrition status assessment and another 10 participants for not completing cognitive assessment. The data was collected using face to face and one-on-one personal interviews conducted by medical students who were trained to interview study subjects and collect the questionnaire data. Other anthropometric and bioimpedance measurements were collected by trained technicians.

### Sarcopenia evaluation

Sarcopenia was measured according to the AWGS 2014 diagnostic criteria by assessing muscle mass, muscle strength, and physical performance [33]. Bioelectric Impedance Analysis (BIA) was performed to determine muscle mass using the INbody770 body composition instrument [34]. The cut-off value for the appendicular skeletal muscle mass index (ASMI) was 7.0 kg/m^2^ in men and 5.7 kg/m^2^ in women [33].

Grip strength was measured with a grip dynamometer (EH101; Camry, Zhongshan, China). During the grip strength test, subjects held the grip dynamometer with their dominant hand, stood upright, kept their feet separated (shoulder-width apart), and let their arms droop naturally. The test was performed twice independently and the largest value was used for the final analysis. The cut-off grip strength value was 26 kg in men and 18 kg in women [33].

Physical performance was determined by measuring gait speed with an infrared sensor. The acceleration phase was strictly excluded from the walking time. During the test, subjects wore common shoes and could use mobility aids, but were not assisted by others. The cut-off value of gait speed was 0.8 m/s^13^.

### Evaluation of other clinical parameters

The baseline demographic information included (1) General personal data: age, gender, ethnicity (Han, Zang, Qiang, Yi and others), educational level, and occupation; (2) Lifestyle characteristics: tea drinking, alcohol drinking, and smoking. Anthropometric measurements included height, weight, and body mass index (BMI). Sleep quality was assessed using Pittsburgh sleep quality index (PSQI). PSQI scores >5 were considered as characteristic of poor sleep quality [35]. Cognitive status was measured using the 10-item Short Portable Mental Status Questionnaire (SPMSQ) [36]. Higher SPMSQ scores indicated lower cognitive ability. Depressive symptoms were assessed using 15-item Geriatric Depression Scale (GDS-15) and patients with GDS-15 scores ≥5 were classified as depressed [37]. Anxiety status was assessed using the Generalized Anxiety Disorder (GAD-7) questionnaire and patients with GAD-7 scores ≥5 were considered as those with anxiety [38]. Nutrition status was graded using the Mini Nutrition Assessment-Short Form (MNA-SF) scale; MNA-SF scores from 0~7 indicated malnutrition status, 8~11 indicated malnutrition risk, 12~14 indicated good nutrition status [39]. Patients self-reported any medical history of chronic disease such as hypertension, osteoarticular disease, coronary heart disease, lung disease, diabetes mellitus, tumors, and others.

### Statistical analysis

Statistical analysis was performed using the R software (version 4.0.2). Kolmogorov-Smirnov test was used to determine normalized distribution of variables. The baseline data are presented as means± standard deviation (SD) or frequencies. The differences between groups were analyzed by one-way analysis of variance (ANOVA) for continuous variables and chi squared test for categorical variables. The association between cognitive score and sarcopenia was analyzed by binary regression using four separate models in which cognitive decline was plotted as the predictor variable and sarcopenia categories were plotted as the outcome variables. The four models were as follows: (1) Model 1 adjusted by sex, gender, and ethnic groups; (2) Model 2 adjusted by Model 1 + life styles (smoking, drinking alcohol and drinking tea), and sleep quality; (3) Model 3 adjusted by Model 2 + chronic disease comorbidity, depression and anxiety; (4) Model 4 adjusted by Model 3 + nutrition status. The role of nutrition status in cognitive decline and sarcopenia was analyzed using the Mediation package in R (version 4.0.2) [40]. Mediation hypotheses were adjusted for age, sex, and ethnicity using bias-corrected bootstrap method with 4023 samples to calculate confidence intervals (95%). P < 0.05 was considered statistically significant. The effect was considered indirect if the confidence interval did not include zero. The SEM pathway analysis was performed with the SEM package in R (version 4.0.2) [41].
